The article "Effects of Combined Cognitive and Exercise Interventions on Poststroke Cognitive Function: A Systematic Review and Meta-Analysis" was published in 2021. Journal: Biomed Res Int.

# Effects of Combined Cognitive and Exercise Interventions on Poststroke Cognitive Function: A Systematic Review and Meta-Analysis

**DOI:** 10.1155/2021/4558279

**Published:** 2021-11-17

**Authors:** Ruifeng Sun, Xiaoling Li, Ziman Zhu, Tiancong Li, Wenshan Li, Peiling Huang, Weijun Gong

**Affiliations:** ^1^Beijing Rehabilitation Medicine Academy, Capital Medical University, Beijing, China 100144; ^2^Department of Neurological Rehabilitation, Beijing Rehabilitation Hospital, Capital Medical University, Beijing, China 100144

## Abstract

**Objective:**

We investigated combined cognitive and exercise interventions in the literature and summarized their effectiveness in improving poststroke cognitive impairment (PSCI). *Data Sources*. Electronic databases and trial registries were searched from their inception until July 2020. *Study Selection*. Trials were collected with the following study inclusion criteria: (1) patients over 18 years of age who were diagnosed with PSCI; (2) combined cognitive-exercise interventions, regardless of the order of the two types of interventions or whether they were administered simultaneously; (3) any control group studied at the same time that was deemed acceptable, including no intervention/routine care, delayed intervention, sham intervention, and passive training; (4) the use of any validated cognitive neuropsychological test to evaluate cognitive function; and (5) clinically administered random trials with controls. *Data Extraction*. Five randomized controlled trials met the inclusion criteria. Two reviewers independently assessed the eligibility of the full texts and methodological quality of the included studies using the Cochrane risk of bias tool. Inconsistent results were resolved by additional discussion or decided by a third examiner, if necessary. *Data Analysis*. Meta-analysis demonstrated that the combined interventions had a significant effect on executive function and working memory [Stroop test (time), standardized mean difference (SMD) = 0.42, 95% confidence interval (CI): 0.80–0.04, *p* = 0.02; Trail Making Test, SMD = 0.49, 95% CI: 0.82–0.16, *p* = 0.004; Forward Digit Span Test, SMD = 0.91, 95% CI: 0.54–1.29, *p* ≤ 0.001]. While it was impossible to conduct a meta-analysis of global cognitive function and other cognitive domains, individual experiments demonstrated that the combined interventions played a significant role in global cognition, reasoning ability, logical thinking, and visual-spatial memory function.

**Conclusions:**

Our analyses demonstrated that the combined interventions had a significant effect on the improvement of PSCI, particularly in terms of executive function. However, the moderate risk of bias in the included trials and the small number of relevant studies indicated a need for more uniform diagnostic and evaluation criteria, and larger trials would provide stronger evidence to better understand the effectiveness of the combined interventions. This trial is registered with trial registration number INPLASY202160090.

The article "Effects of Combined Cognitive and Exercise Interventions on Poststroke Cognitive Function: A Systematic Review and Meta-Analysis" was published in 2021. Journal: Biomed Res Int.

## 1. Introduction

Strokes are a serious public health problem, with over 795,000 cases recorded in the United States every year. On average, one person has a stroke every 40 s, and one person dies of a stroke every 4 min [1]. China has the highest incidence of strokes worldwide. In 2016, the incidence of ischemic strokes reached 277/100,000, and the incidence of hemorrhagic strokes reached 126/100,000. Strokes are currently the second leading cause of disability, behind only ischemic heart disease. In 2016, more than 80 million people worldwide suffered from stroke sequelae [2]. Strokes are the second most common cause of dementia. Poststroke cognitive impairment (PSCI) refers to a series of syndromes that meet the diagnostic criteria of cognitive impairment within 6 months after a stroke. This definition emphasizes the potential causality and importance of clinical management between strokes and cognitive impairment, including cognitive impairment caused by strokes resulting from key infarction, multiple infarctions, subcortical ischemic infarction, and cerebral hemorrhage. In this case, cognitive impairment includes executive dysfunction, memory dysfunction, attention disorder, orientation disorder, and perception disorder [3]. Previous studies have demonstrated that more than 32% of stroke survivors show cognitive dysfunction [4]. According to the Mini-Mental Status Examination (MMSE) standard assessment, the incidence of cognitive dysfunction within 3 months of a stroke is 24%–39% in the United Kingdom and Switzerland [5]. A large-scale, multicenter cohort study in South Korea recruited 620 patients with ischemic strokes as assessed by the MMSE and found that the prevalence of PSCI reached 69.8% in patients within 3 months of the stroke [6]. PSCI is associated with decreased self-care ability and quality of daily life, the accelerated decline of body functions, and an increased risk of disability and death.

Several strategies to improve cognition have been explored in both healthy individuals and patients with Alzheimer's disease. Extensive studies have demonstrated that cognitive training (including cognitive-behavioral training and computer-assisted cognitive training) and exercise training (including aerobic exercise and resistance exercise) can effectively improve cognitive function [7–10]. A meta-analysis indicated that for PSCI patients, exercise training can positively impact global cognition and that a combination of aerobic exercise and strength training produces the greatest cognitive benefits. Exercise can also improve cognitive function in patients with chronic stroke. It provides a moderate improvement in treatment speed, and it can be used as an intervention strategy to improve PSCI [11]. Cognitive training is also essential for treating PSCI and is primarily divided into compensation training strategies and direct repair cognitive training [12]. Direct repair cognitive training includes practical exercises, memory training (such as reciting acronyms or songs), and computer-aided cognition training. A systematic review of eight studies conducted by Law et al. demonstrated that the combined interventions could effectively improve cognitive function in the elderly with or without cognitive impairment [13]. However, there is not a conclusion on the role of cognitive impairment in stroke patients. This study mainly intended to review the evidence and evaluate the impact of combined interventions on PSCI.

The article "Effects of Combined Cognitive and Exercise Interventions on Poststroke Cognitive Function: A Systematic Review and Meta-Analysis" was published in 2021. Journal: Biomed Res Int.

## 2. Methods

### 2.1. Inclusion Criteria

Trials were included for this review if they met the following criteria: (1) research subjects—patients over 18 years of age who were diagnosed with PSCI, excluding other types of vascular cognitive impairment and various nonvascular cognitive impairments related to stroke; (2) intervention—combined cognitive-exercise intervention that included both cognition and exercise training, regardless of their order or whether they were administered simultaneously (for example, memory training after walking on a treadmill or while walking on a treadmill); (3) comparison—any control group studied at the same time was deemed acceptable, including no intervention/routine care, delayed intervention, sham intervention, and passive training; (4) result—the use of any validated cognitive neuropsychological test to evaluate the cognitive function as a primary or secondary result; and (5) research design—clinically administered random trials with controls.

### 2.2. Exclusion Criteria

Trials were excluded if they met the following criteria: (1) nonintervention research; (2) theoretical articles or descriptions of treatment methods; (3) review articles; (4) unpublished studies, abstracts, or papers; (5) articles that did not fully explain the intervention measures; (6) non-peer-reviewed articles or book chapters; and (7) non-English articles.

### 2.3. Search Strategy

We systematically searched the PubMed, EMBASE, and Cochrane Library electronic databases, clinical trial registration websites, and clinical randomized controlled trials published in peer-reviewed journals from the earliest available record until July 2020. We used the following keyword combinations to find relevant articles: (rehabilitation OR habilitation OR combine^∗^ interventions OR dual-task OR multi-modal) OR (exercise OR physical activity OR resistance training OR endurance training) AND (cognitive function OR cognition OR attention OR memory OR executive function OR neuropsychological test) AND (dementia^∗^, vascular OR stroke OR cerebrovascular accident OR brain ischemia OR poststroke OR post-stroke OR vascular dementia^∗^ OR vascular cognitive impairment).  Table 1 presents examples of the PubMed search methods. When possible, all search keywords were combined with medical MeSH words and free words to identify relevant research. EndNote X9 was used to store and sort the retrieved randomized controlled trials and delete duplicate documents. Two individuals independently screened titles and abstracts according to the predefined inclusion criteria. The full text of all trials that met the inclusion criteria was searched based on the title and abstract, which was the basis for identifying the articles included in this study. Inconsistent results were determined by additional discussion or decided by a third examiner, if necessary.

The article "Effects of Combined Cognitive and Exercise Interventions on Poststroke Cognitive Function: A Systematic Review and Meta-Analysis" was published in 2021. Journal: Biomed Res Int.

The meta-analysis was performed in accordance with the PRISMA guidelines, and the checklist was completed (registration number: INPLASY202160090).

### 2.4. Data Extraction

The Cochrane data extraction form was used to extract data according to the following parameters: (1) basic information—research title, number, source of publication, and research funding; (2) inclusion/exclusion criteria—research design, population sample, intervention type, implementation site, and outcome indicators; (3) research methods and characteristics—research period, sample size, generation and concealment of distribution sequence, blind method, and other related bias problems; (4) subject characteristics—number of subjects, diagnostic criteria, age, gender, and country; (5) intervention/comparison—grouping, specific intervention measures, duration, frequency, intensity, and completeness of the intervention process; (6) outcome measurement—all relevant cognitive results and measurement tools and the measurement time point of outcome indicators; and (7) conclusion—two personnel that cross-checked to extract data for each trial. Inconsistent results were determined by additional discussion or decided by a third examiner, if necessary.

### 2.5. Literature Quality Evaluation

The Cochrane risk of bias assessment tool was used to independently assess the risk of bias in the included trials. The assessment scope included the following parameters: random sequence generation, allocation concealment, blinding, incomplete data, and selective reporting. Each part was classified into three categories: low-risk, unclear, and high-risk. Each trial was classified using the following criteria: low risk of bias (all criteria were rated as low-risk); medium risk of bias (one standard was rated as high-risk, or two criteria were rated as unclear); and high risk of bias (multiple criteria were rated as high-risk, or more than two were rated as unclear). Two examiners conducted independent evaluations, and inconsistent results were resolved by additional discussion or decided by a third examiner, if necessary.

The article "Effects of Combined Cognitive and Exercise Interventions on Poststroke Cognitive Function: A Systematic Review and Meta-Analysis" was published in 2021. Journal: Biomed Res Int.

### 2.6. Data Analysis

Cognitive results were grouped according to the cognitive domains that were evaluated (such as global cognition, executive function, and memory), and the baseline–endpoint difference of neuropsychological tasks was used to conduct a meta-analysis of related cognitive domains. The following correlation coefficient equation was used to calculate the baseline–endpoint SD change:

(1) $$\begin{array}{c} {\text{SD}}_{\frac{1}{\text{change}}}=\sqrt{{\text{SD}}_{\frac{1}{{\text{baseline}}^{2}}}}+{\text{SD}}_{\frac{1}{{\text{final}}^{2}}}-\left(2\times R_{1}\times {\text{SD}}_{\frac{1}{\text{baseline}}}\times {\text{SD}}_{\frac{1}{\text{final}}}\right),\text{R}1=0.5. \end{array}$$

Review Manager (version 5.2) was used for the meta-analysis and data processing. The standardized mean difference (SMD) of continuous variables and a 95% CI were used for quantification. The heterogeneity between the experimental design schemes was unclear; so the fixed effects model was chosen. *I*^2^ statistics measured heterogeneity.

## 3. Results

### 3.1. Search Results

We obtained 1,198 related references by searching the electronic databases. Duplicates were removed, and the titles and abstracts were examined according to the pre-set inclusion criteria. Twenty-eight full references were retained, and we conducted a detailed review of each paper. A total of 22 trials did not meet the preset inclusion criteria. Reasons included nonrandomized control trials (*n* = 1), irrelevant interventions (*n* = 3), ongoing trials (*n* = 13), research protocols (*n* = 4), and unevaluated cognitive outcomes (*n* = 1). Six randomized control trials met the preset inclusion criteria, and one study did not obtain the original trial data [14]. Therefore, a total of five trials were included in this study.

### 3.2. Research Characteristics

The five randomized controlled trials included in this study were published between 2015 and 2019 (Table 2). A total of 362 participants (58.2% male) were assigned to the corresponding intervention group or the control group during the same period, while the study sample scale was between 25 and 225. All test subjects met the PSCI diagnostic criteria. In one trial, the inclusion criteria of the test population stipulated that patients must have had stroke less than 6 months prior [15], while the remaining four subjects were all PSCI patients with an onset time of stroke more than 6 months prior. In two of the trials, the subjects were divided into a cognitive-exercise combined group, a cognitive training group, an exercise training group, and a control group, all of which included follow-up results [15, 16]. In one trial, evaluations were conducted twice after interventions at 3 and 6 months [17]. The test sites included two at the rehabilitation hospital [16, 18], two at the hospital rehabilitation center [15, 19], and one in the community [17]. The total number of interventions in each study ranged from 18 to 48, the training frequency was 2–3 times a week, and the training duration was 30–60 min.

The article "Effects of Combined Cognitive and Exercise Interventions on Poststroke Cognitive Function: A Systematic Review and Meta-Analysis" was published in 2021. Journal: Biomed Res Int.

One trial assessed the effects of simultaneous cognitive-exercise intervention on cognitive function [18], and the other four assessed the effects of sequential cognitive-exercise intervention on cognitive function [15–17, 19]. For three trials, the cognitive-exercise intervention included aerobic exercise, resistance exercise, or balance exercise with computer-aided cognitive training [15, 16, 19]. One trial included aerobic exercise, resistance exercise, or balance exercise with entertainment and social activities designed to improve planning, logic, decision-making, and learning ability [17]. One trial included simultaneous cognitive-exercise intervention as balanced movement+cognitive-behavioral training (including reverse recitation, forward retelling, reverse retelling, word association, calculation, attention, and anti-interference ability training) [18] (Table 3).

### 3.3. Cognitive Outcome Evaluation

Three trials [15, 17, 18] investigated the effect of the combined interventions on subdomains of executive function (including selective attention, conflict resolution, and anti-interference ability), attention maintenance, cognitive flexibility, working memory, and memory span. The Stroop test, Trail Making Test, and Digit Span Test were used as evaluation tools. The Stroop test was mainly used to assess conflict inhibition, cognitive control, response flexibility, and selective attention; the Trail Making Tests (TMT-A, TMT-B) were used to examine the patient's ability to recognize the symbolic meaning of numbers and letters and connect them in order. To assess attention span and cognitive flexibility in cognitive function, the Digit Span Test was performed. The Digit Span Test is a digital memory test used to evaluate working memory, memory span, and attention to auditory stimuli, regardless of age and education limits. One study used Raven's Progressive Matrices to assess observation, reasoning, and logical thinking skills [16]. Only one trial evaluated the results of cognitive neuropsychology involving global cognitive function [19]. The MoCA scale was used as the primary metric of cognitive function, while the secondary outcome indicators used the Wechsler Memory Scale-III (WMS-III) Spatial Span to evaluate visual-spatial memory function and the WMS-III Verbal Pair to evaluate verbal learning and memory function.

The article "Effects of Combined Cognitive and Exercise Interventions on Poststroke Cognitive Function: A Systematic Review and Meta-Analysis" was published in 2021. Journal: Biomed Res Int.

### 3.4. Literature Quality Evaluation

The quality of the research varied in the included trials (Figure 1). One trial had a low overall risk of bias [18], three trials had a moderate overall risk of bias, and one trial had a high overall risk of bias [19].

### 3.5. The Impact of the Combined Interventions on Cognitive Outcomes

Three trials evaluated the impact of the combined intervention on the results of the Stroop test, Trail Making Test, and Digit Span Test. There were a total of 69 people in the test group and 76 people in the control group in these three trials.

#### 3.5.1. Stroop Test

Liu et al. [17] and Wang et al. [15] compared the time required to complete the Stroop test before and after intervention; the less time it took, the stronger the selective attention, conflict resolution, and anti-interference ability. Park and Lee [18] measured the number of words correctly read in the Stroop test within 120 s. The more the number of correct words that were read, the better the cognitive function. Due to different measurement methods and indicators, only the first two groups were combined and analyzed during data analysis. There was no evidence of heterogeneity in any measurements (*I*^2^ = 0%). The statistical results demonstrated that combined interventions can significantly improve the Stroop test_(time)_ score (SMD = −0.42, 95% CI: −0.80 to −0.04, *p* = 0.02, Figure 2). Park et al. measured the number of words and colors correctly identified in 120 s, and the results showed significant improvement before and after the intervention. When a comparative evaluation was performed with the control group, the number of color words the participants were able to correctly identify within 120 s improved significantly (*p* = 0.023). On the Stroop word items, the number of correct words in the dual-task group increased by 14.8 on average, while that in the control group decreased by 0.1 on average. On the Stroop color items, the number of correct colors increased by 18.35 in the dual-task group and by 0.65 in the control group.

The article "Effects of Combined Cognitive and Exercise Interventions on Poststroke Cognitive Function: A Systematic Review and Meta-Analysis" was published in 2021. Journal: Biomed Res Int.

#### 3.5.2. Trail Making Test

Three trials [15, 17, 18] assessed the changes in the time required to complete the online test before and after the intervention. Park et al. assessed the results of the TMT-A and B. In this study, we only combined and analyzed the TMT-B results and found that the shorter the test time, the better the attention span and cognitive flexibility. Larger differences indicated better intervention effects. The results of the combined data analysis found no evidence of heterogeneity in any of the measurements (*I*^2^ = 0%). The statistical data of the two groups revealed a significant effect between combined intervention and the control group. Combined interventions can shorten the duration of the TMT (SMD = −0.49, 95% CI: −0.82 to −0.16, *p* = 0.004, Figure 3). Liu et al. showed that the combined intervention significantly slowed down the decline of the completion speed of TMT-B, with an average reduction of 0.4 s in the combined intervention group and an average increase of 28.9 s in the control group. Park et al. and Wang et al. showed that the completion time of TMT-B was significantly shortened in the combined intervention group.

#### 3.5.3. Digit Span Test

Park and Lee [18] and Wang et al. [15] measured the changes in the length of the Digit Span Test forward and backward before and after the intervention. According to the sequence of numbers they heard, Liu et al. [20] had the subjects repeat a gradually increasing sequence of random numbers in order or reverse order. The tester then subtracted the forward test score from the reverse test score to obtain a working memory index; the smaller the difference score, the better the memory performance. The first two trials were different from subsequent measurements. Wang et al. only evaluated the results of a Digit Span Test forward and backward; so, only the digital results of the first two trials were combined and analyzed. Our results demonstrated that the combined interventions had a significant impact (Forward Digit Span Test SMD = 0.91, 95% CI: 0.54 to 1.29, *p* ≤ 0.00001, Figure 4). The results of the Digit Span Test obtained by Liu et al. showed that the combined intervention group had a statistically significant difference in working memory compared with control group (*p* = 0.04).

The other two trials were not included in the meta-analysis due to differences in neurocognitive psychology assessment methods. Ploughman et al. [16] conducted Raven's Progressive Matrices test and found that the combined intervention yielded statistically significant differences in reasoning ability, observation ability, and the logical thinking ability of PSCI patients [*F*(3, 48) = 4.03, *p* = 0.012]. Yeh et al. [19] reported that the combined intervention significantly affected global cognitive MoCA [*F*(1, 27) = 5.236, *p* = 0.03] and visual-spatial memory function as measured by the WMS-III Spatial Span [*F*(1, 27) = 7.193, *p* = 0.012]. After intervention, the average MoCA score of the combined intervention group increased by 4.86 points, while that of the control group increased by only 2 points. However, there was no significant difference in the memory function of the language learning WMS-III Verbal Pair [*F*(1, 27) = 0.223, *p* = 0.641].

The article "Effects of Combined Cognitive and Exercise Interventions on Poststroke Cognitive Function: A Systematic Review and Meta-Analysis" was published in 2021. Journal: Biomed Res Int.

## 4. Discussion

In this study, we examined the effectiveness of combined interventions to improve PSCI. Five studies met the inclusion criteria and were included in this review. All subjects were PSCI patients. One of the studies included patients whose stroke had occurred less than 6 months prior to the study, and the remaining subjects from the other four studies all had strokes more than 6 months prior to the study. One study was published in 2015, and the other four were published in 2019. This suggested that research assessing how combined interventions affect cognitive function after a stroke was still in its early stages and that the potential benefits of combined interventions were beginning to attract the attention of researchers. The studies in this review were mainly from developed countries, including China. The overall quality of the trials was uneven, with most trials having a moderate or high risk of bias. The lack of common results and the insufficient number of trials limited the robustness of the meta-analysis. More research is needed to obtain sufficient evidence before a reliable conclusion can be drawn that combined interventions can effectively improve cognitive function, particularly executive function, in patients with PSCI. Three studies found that combined intervention could significantly improve selective attention, conflict resolution, anti-interference ability, attention maintenance, cognitive flexibility, working memory, and memory span. This review provides specific research attributes that will be of use for future research.

### 4.1. Research Status in the Past Reviews

A recent review systematically evaluated the effect of combined interventions on the cognitive function of elderly individuals both with and without cognitive impairment [13]. It supported the finding that combined interventions could improve cognitive function in healthy elderly individuals and could significantly improve cognitive function in patients with cognitive dysfunction. However, there was a lack of comparison with a positive control group, and the available evidence was limited. Therefore, the data were insufficient to conclude that combined interventions would result in cognitive improvement for elderly individuals with cognitive impairment. Another systematic review evaluated the effects of an exercise intervention on the cognitive function of PSCI patients [11] and found that there was a significant improvement with small to moderate positive effects in the chronic stroke stage. There was no relevant summary assessing the impact of the combined intervention on PSCI. This review synthesized quantitative data from intervention trials that evaluated the impact of combined intervention on cognitive impairment in patients with stroke. The current research was in its primary stage, the available data were limited, and the evaluation indicators were not uniform. Therefore, only a small number of studies were included in this meta-analysis. This review provided supporting data for the effects of the combined intervention on cognitive function in patients with strokes. After performing a Stroop test, a Trail Making Test, and a Digit Span Test, the intervention group showed significant improvements in executive function and memory. Our findings indicated that combined interventions significantly affected the executive function. The combined interventions also showed positive effects on global cognition, logical thinking, attention, and memory. However, these conclusions were drawn based on a single study, and no meta-analysis was performed.

The article "Effects of Combined Cognitive and Exercise Interventions on Poststroke Cognitive Function: A Systematic Review and Meta-Analysis" was published in 2021. Journal: Biomed Res Int.

### 4.2. Experimental Design

There was no unified standard in the design of the studies for this review, and these differences in trial design highlighted the need for additional research. The intervention time of some of the trials was very short (30 min/time), and the total number of interventions for all included trials ranged from 18 to 48. A previous meta-analysis [21] evaluated the relationship between exercise and cognition, finding that interventions that lasted for 6 months or longer are more likely to significantly influence cognition than shorter interventions. Another meta-analysis found no positive correlation between intervention duration and the impact of cognitive intervention on patients with mild cognitive impairment (MCI), indicating that longer periods of intervention did not necessarily produce better results [20]. Different types of interventions were used in the trials included in this study, which could affect the results. Previous studies have demonstrated that a combination of aerobic and resistance training could have greater cognitive benefits compared with aerobic or resistance training alone [10, 22], while a meta-analysis by Wang et al. showed that high-intensity training and frequent resistance exercise could be the most effective method for improving the global cognition of adults with MCI [23]. In addition, intervention measure compliance rates during trial design were rarely reported. Therefore, when interpreting trial results, it is important to provide compliance data that could affect the magnitude of the treatment effect and provide guidance on the acceptability of interventions [24].

The article "Effects of Combined Cognitive and Exercise Interventions on Poststroke Cognitive Function: A Systematic Review and Meta-Analysis" was published in 2021. Journal: Biomed Res Int.

### 4.3. Intervention Sequence

In the combined cognitive-exercise training, the implementation time of the two types of training could affect the intervention results differently. Cognitive and exercise training could be performed simultaneously or sequentially, and the sequence of cognitive training and exercise training could impact the intervention results. In addition to the training sequence, whether the training is continuous or intermittent and the length of the interval could impact cognitive function. Legault et al. found that exercise training after cognitive training did not significantly improve the patient's condition [25]. However, Oswald et al. showed that exercise training prior to cognitive training could produce positive effects [26]. Barcelo et al. demonstrated that simultaneous exercise–cognitive training combining aerobic training with cognitive and memory training was related to cognitive improvement in healthy elderly people [27]. However, it was unclear whether this conclusion was applicable to PSCI patients. Animal studies have shown that exercise promotes nerve regeneration in the brain and improves learning ability [28]. Neuroimaging studies of patients with cognitive impairment have found that compensatory recruitment of new brain cells was observed when completing complex tasks [29]. Some researchers proposed that the physical portion of the combined intervention training increased the brain's neurogenesis potential when exposed to complex cognitive tasks [30]. Exercising before cognitive training also appeared to better prepare the brain for compensatory recruitment in subsequent cognitive training. A meta-analysis of the effects of combined cognitive-exercise training (including simultaneous training and sequential training) on the cognitive function of elderly people conducted by Zhu et al. suggested that the combined intervention could improve the cognitive function of the elderly compared with the control group and the exercise group, but the results were not statistically significant compared with the cognitive training group. The subgroup analysis suggested that the effect of simultaneous cognitive and exercise training was higher than that of sequential training. However, these results were not statistically significant compared with the cognitive training group, though the subgroup analysis suggested that simultaneously treating patients with cognitive-exercise intervention had better effects than sequential training [31].

The article "Effects of Combined Cognitive and Exercise Interventions on Poststroke Cognitive Function: A Systematic Review and Meta-Analysis" was published in 2021. Journal: Biomed Res Int.

### 4.4. Limitations

The primary limitations of this review were the lack of common outcome metrics and the small number of studies. The use of different kinds of cognitive tasks to measure the same cognitive functions made it difficult to directly compare the results of the different experiments. Even if the same cognitive task was used for evaluation, there were inconsistencies in the data reporting methods, the neuropsychological tests varied in form and complexity, and there was a lack of guidelines for evaluators. These factors made it difficult to compare and analyze different trials. Additionally, different trials focused on different cognitive functions, making it difficult to merge and analyze data. All of this must be considered when assessing the conclusion that combined interventions can significantly improve cognitive function in stroke patients.

### 4.5. Implications for Future Research

The duration of intervention training in the trials varied, as did the training methods. Subsequent trial design should explore the intervention duration and intervention mode and assess training compliance. The lack of homogeneity among the cognitive results in the current trials made it difficult to compare the results. Future studies should establish a core set of guidelines to standardize the evaluation of cognitive outcomes in PSCI research. In addition to the executive function assessed in this review, research should also focus on global cognitive function and cognitive domains of important clinical significance, such as visual and language memory, attention span, and processing speed. Therefore, it is very important to identify the cognitive domains and neuropsychological tests that are most sensitive to cognitive decline after stroke, as well as the cognitive domains and neuropsychological tests that are most sensitive to changes in nondrug interventions (such as exercise and cognitive training). In addition, previous research suggested that exercise and cognitive training could improve the cognitive ability of elderly individuals by increasing neurotrophic factors and neurotransmitters, increasing cerebral blood flow, reducing inflammation, and changing the brain structure [32–35]. Future research should focus on elucidating the factors related to exercise and cognitive training in terms of brain biomarkers and neuroimaging in PSCI patients. More well-designed studies are needed, especially ones focusing on comparative control and population screening, selection of outcome indicators, training sequence, intervention time, and results, to reveal the different effects of cognitive-exercise combined training on PSCI. In the absence of a cure for cognitive impairment or dementia, further research efforts are needed to explore the potential benefits of this new intervention model that could help delay or reverse cognitive impairment.

The article "Effects of Combined Cognitive and Exercise Interventions on Poststroke Cognitive Function: A Systematic Review and Meta-Analysis" was published in 2021. Journal: Biomed Res Int.

## 5. Conclusion

This study found that cognition–exercise combined interventions had significant benefits for the global cognitive function, executive function, attention span, and memory function of PSCI patients. However, the number of trials assessing these variables was limited. Fortunately, there has been an increase in studies assessing these factors in recent years. This subject is worthy of further research. Besides comparing the combined intervention and the control group, it is also necessary to explore the impact of the combined intervention and single-task training on cognition and compare the effects of cognitive-exercise sequential training with those of simultaneous training.

## Figures and Tables

**Figure 1:** Risk of bias assessment of included trials.

**Figure 2:** Trial level data, effect estimates, and forest plot for the effects of combined interventions on the Stroop test (time).

**Figure 3:** Trial level data, effect estimates, and forest plot for the effects of combined interventions on the Trail Making Test.

**Figure 4:** Trial level data, effect estimates, and forest plot for the effects of combined interventions on the Forward Digit Span Test.

**Table 1:** Search strategy.

1# “Rehabilitation”[MeSH]	2# (((Habilitation[Title/Abstract]) OR (combine∗ interventions[Title/Abstract])) OR (dual-task[Title/Abstract])) OR (multi-modal[Title/Abstract])
3# 1# AND 2#	
4# “Exercise”[MeSH]	5# (((((((((((((((physical activity[Title/Abstract]) OR (resistance training[Title/Abstract])) OR (endurance training[Title/Abstract])) OR (Exercise∗[Title/Abstract])) OR (Physical Activity∗[Title/Abstract])) OR (Activity∗, Physical[Title/Abstract])) OR (Exercise∗, Physical[Title/Abstract])) OR (Physical Exercise∗[Title/Abstract])) OR (Acute Exercise∗[Title/Abstract])) OR (Exercise∗, Acute[Title/Abstract])) OR (Exercise∗, Isometric[Title/Abstract])) OR (Isometric Exercise∗[Title/Abstract])) OR (Exercise∗, Aerobic[Title/Abstract])) OR (Aerobic Exercise∗[Title/Abstract])) OR (Exercise Training∗[Title/Abstract])) OR (Training∗, Exercise[Title/Abstract])
6# 4# AND 5#	
7# “Cognition”[MeSH]	8# (((((((((((Cognitive Function∗[Title/Abstract]) OR (Function∗, Cognitive[Title/Abstract])) OR (Focus of Attention[Title/Abstract])) OR (Attention Focus[Title/Abstract])) OR (attention[Title/Abstract])) OR (memory[Title/Abstract])) OR (executive function[Title/Abstract])) OR (Executive Functions[Title/Abstract])) OR (Function∗, Executive[Title/Abstract])) OR (Executive Control∗[Title/Abstract])) OR (cognitive function[Title/Abstract])) OR (neuropsychological test[Title/Abstract])
9 # 7# AND 8#	
10# ((((stroke[Title/Abstract]) OR (cerebrovascular accident[Title/Abstract])) OR (brain ischemia[Title/Abstract])) OR (poststroke[Title/Abstract])) OR (post-stroke[Title/Abstract])	
11# 3# OR 6# AND 9# AND 10#	

The article "Effects of Combined Cognitive and Exercise Interventions on Poststroke Cognitive Function: A Systematic Review and Meta-Analysis" was published in 2021. Journal: Biomed Res Int.

**Table 2:** Baseline characteristics of included trials.

Author	Year	Country/region	Intervention cycle (number of times)	Grouping	Baseline age (years)	Baseline number	Drop-off number	Male composition ratio (%)	MMSE	MoCA
Liu	2015	Canada	48	INT	62.90 (12.10)	25	1	60		24.80 (2.60)
				D-INT	66.90 (9.00)					21.80 (6.90)

Park	2019	South Korea	18	DT	56.30 (7.14)	30	0	69.2	26.50 (2.52)	
				COT	59.75 (7.75)				25.60 (2.91)	

Ploughman	2019	Canada	30	Aerobic+COG	62.10 (14.20)	52	0	36		23.30 (7.50)
				Aerobic+games	58.40 (11.70)					24.90 (4.80)
				Activity+COG	63.90 (8.50)					24.90 (4.70)
				Activity+games	69.70 (8.90)					21.90 (5.40)

Wang	2019	China	36	TT	66.68 (2.44)	225	46	55.6	17.45 (5.62)	
				PE	65.12 (2.56)				16.82 (5.83)	
				CT	67.51 (2.24)				15.69 (6.21)	
				CO	64.36 (2.31)				16.79 (6.35)	

Yeh	2019	Taiwan	36	Sequential group	50.63 (3.99)	30	0	70	25.80 (0.92)	20.07 (1.08)
				Control group	60.21 (3.10)				24.57 (0.78)	18.79 (1.36)

INT: intervention; D-INT: delayed intervention; DT: dual-task training; COT: conventional occupational therapy; COG: cognitive training or games; TT: combined intervention of physical exercise and cognitive training; PE: physical exercise; CT: cognitive training; CO: control group; MMSE: Mini-Mental State Examination; MoCA: Montreal Cognitive Assessment.

**Table 3:** Intervention characteristics of included trials.

Author	Year	Country/region	Intervention times	Type of exercise training	Type of cognitive training	Frequency	Duration (min)
Liu	2015	Canada	48	Aerobic+resistance+balance training	Collective activity for cognitive training	3/W	60
Park	2019	South Korea	18	Balance training	Cognitive training	3/W	30
Ploughman	2019	Canada	30	Aerobic exercise	Computerized dual-n-back training	3/W	20–30
Wang	2019	China	36	Aerobic+resistance+balance training	Computer-based cognitive training	3/W	50
Yeh	2019	Taiwan	36	Aerobic exercise	Computer-based cognitive training	2–3/W	60

## Abbreviations

PSCI: Poststroke cognitive impairment
SMD: Standardized mean difference
CI: Confidence interval
MMSE: Mini-Mental State Examination
SD: Standard deviation
MoCA: Montreal Cognitive Assessment
MCI: Mild cognitive impairment.
